# Integrating Mental Health Education into French Teaching in University Based on Artificial Intelligence Technology

**DOI:** 10.1155/2022/1046813

**Published:** 2022-09-12

**Authors:** Jingli Zhao

**Affiliations:** Shanghai University of International Business and Economics, Shanghai 201620, China

## Abstract

In recent years, there has been a lot of news about college students committing suicide. In the university stage students, self-esteem is stronger and more sensitive, and the ability to withstand pressure is weak. At the same time, college students are in a key stage of mental health development. School education to a certain extent for the cultivation of students' mental health has a crucial impact. In our country, it is undoubtedly the main way to infiltrate mental health education through subject knowledge teaching. French teaching is a good way to infiltrate mental health education. In the learning practice, the improvement of students' mental health levels can strengthen their interest in French learning. Based on this, this paper, from the perspective of French teaching, carries out the infiltration of mental health education in French teaching classes in universities and promotes the cultivation of students' learning abilities and the development of mental health. This paper mainly studies the feature extraction of mental health data, tries to use the optimized BP (backpropagation) neural network to infiltrate the mental health model of college students, and describes the differences in mental health among students. Finally, the results are applied to French teaching in universities, and a good teaching effect is achieved. Finally, the experimental results show that the infiltration strategy proposed in this study is feasible and effective.

## 1. Introduction

When it comes to health, people used to think that there was no disease in the body and that they could live a long life without seeking medical advice. In the minds of Chinese people, there are still many people who agree with this point of view. As early as the 20th century, related organizations had the world within the scope of the definition of health, the most typical is the world health organization (WHO) definition of the concept of health, which has no exception. It points out that health is where the body does not need to please the medical medicine but also has good mental condition to be able to keep up with the pace of development and trends. In the 1990s, the organization refined the concept, saying that health refers to a person's physical and mental state, as well as his or her mental state, being well adapted to social development. In the context of increasing public attention to their own conditions, it is more acceptable to pay attention to mental health [1, 2]. With the rapid development of China's economy, the spectrum of diseases in the population is also growing. Many psychological diseases appear in the population, these psychological diseases will have a lot of negative effects and have the nature of being universal and harmful. Therefore, mental health has become an important public health issue in China [3, 4].

In fact, in recent years, with the rapid development and transformation of China's economy and society, people's ideas have undergone tremendous changes and intense collisions, resulting in more and more psychological problems. Among them, adolescent mental health has become the focus of our attention. Contemporary teenagers are mostly only children and are in an important period of physical and mental development. They experience an immature big flood clash with social change, then a series of social problems. A lot of minors in getting along with people cannot properly handle interpersonal relationships, self-centeredness, or even bad life habits, losing themselves in the world of the Internet and violence. This has formed a major threat and challenge to the growth of minor students. In the past, emotional disorders and other symptoms that used to occur only in adults have now begun to show a trend in younger people. Many teenagers are also troubled by depression and obsessive-compulsive disorder which can even affect their normal life and studies. At the same time, the relevant survey data shows that nearly 15 percent of middle school students have obvious mental health problems. In addition, there are a number of provinces and cities-related research institutions that have carried out the corresponding investigation and research. Data show that the number of psychological problems in China's teenagers increase year by year [5, 6]. At the same time, various cases caused by the psychological problems of teenagers are often reported in the media. Among them, the events that make countless people feel cold are also torturing people's hearts all at the same time. This judgment reveals and emphasizes the important position and role of youth in national development and national rejuvenation. As a progressive force among young people, young college students play a key role in national development and rejuvenation, which requires them not only to have firm ideals, beliefs, and excellent professional qualities but also to have a mature personality and healthy psychological quality.

Health is one of the most concerning problems in modern society. The health of the people is a sign of the prosperity of society as well as the country. In a modern civilized society, education plays an important role in the cultivation of national health and comprehensive quality, and education has an important impact on people's physical and mental health. In recent years, there has been a lot of news about college students committing suicide. In college stage students' self-esteem is stronger and they are more sensitive and their ability to bear pressure is weak. At the same time, school and society will directly or indirectly affect the physical and mental development of high school students. The majority of students spend the longest time in school each day, except at home. Therefore, school education has a vital impact on students' mental health development. There are many ways to educate students about mental health. For example, in China, psychological courses and counseling rooms are common methods of mental health education. Infiltrating mental health education into subject knowledge is also one of the main ways. The purpose of positive psychology is to make individuals live a happy life. It pays attention to the positive psychological quality of individuals and the development of people's potential. Positive psychological quality is an important research topic in positive psychology, which can not only stimulate individual potential and improve people's happiness but also help to prevent and cure physical and mental diseases [7, 8].

Teaching infiltration in psychological education means that teachers consciously teach the art of psychological guidance to mobilize students' intelligence and nonintelligence factors and integrate the contents of teaching materials into psychological education. In the teaching of the conscious penetration and guidance of students, teachers cultivate their keen observation, stable attention, and abstract thinking ability and help them to establish a scientific attitude and scientific spirit, so as to improve the quality of classroom teaching and promote the overall development of students' psychological counseling activities. The course is taught in class through a case study, group discussion, psychological test, group training, and so on. The psychological education course is a series of teaching activities that promote the development of a student's body and mind by cultivating students' good psychological qualities, and finally, enabling students to develop harmoniously. For middle school students, the realization of mental education is one of the important requirements of quality education. The main difference between the psychological education course and teaching is oneness. Mind education class is a single pure form from the angle of mind education. The maximum use of class time results in a single imparting of mind education knowledge. The infiltration of psychological education into teaching has more advantages, with its flexibility, penetration, persistence, multidisciplinary intersections, and imperceptible effects, which can broaden the teaching way of psychological education and adapt to the existing domestic psychological education teaching objectives [9, 10].

The educational and teaching activities are closely related to the development of a student's personality and psychology, and the school's educational activities are mainly subject-teaching activities. So, the main way to infiltrate schools is to infiltrate the course of subject teaching. This kind of infiltration education approach can not only enable students to acquire knowledge and skills related to the subject but also imperceptibly improve students' psychological quality. In this paper, the author will analyze the necessity and feasibility of infiltrating psychological health education into college French teaching. First, it is the need for the development of The Times to infiltrate French teaching into mental health education. Good psychological quality is the basis of high-quality creative talents, but with the increasingly fierce social competition, college students are under more and more pressure in their studies, life, and other aspects, and mental health problems are increasingly prominent, which are extremely adverse factors for the cultivation of creative talents. It is an extremely efficient way to infiltrate mental health education through French teaching to improve mental health and develop creative thinking [11, 12]. Secondly, psychological health education in French teaching is the need for cultivating students' core quality in the biology subject. Psychological health education in college and French teaching can effectively develop students' core French literacy and improve their mental health. Therefore, school education should not only pay attention to the development of intelligence but also pay attention to the cultivation of students' mental health quality, so as to create favorable conditions for the cultivation of people with core literacy. Thirdly, psychological health education in French teaching is the realistic need to solve students' psychological problems. College is not only the golden period for acquiring knowledge but also the critical period for psychological development. However, considering the tight teaching time and heavy teaching tasks in universities, it is an economical and efficient way to infiltrate mental health education through French teaching classes. Students can obtain French knowledge and skills at the same time. Psychological problems can also be effectively solved.

Mental health development is an eternal topic, and related research is also in progress. However, the academic discussions on mental health education and foreign languages are mostly confined to the perspective of the French subject itself, and there is almost no discussion and analysis from the perspective of French teaching. Therefore, from the perspective of foreign language learning, the infiltration of mental health education into French classrooms can provide new ideas and experiences for later related research and university French teaching. This study will provide some teaching methods that incorporate foreign language learning into the mental health knowledge and education of university students in the teaching of French. For example, there are situational creation methods, cooperative learning methods, and so on. At the same time, French knowledge is taken as a carrier to convey information to students to promote the development of mental health, so as to achieve the goal of promoting the psychological health and harmonious development of school students.

## 2. Related Work

School mental health education in the modern sense originated in developed western countries. The research shows that at present, school mental health education in Britain and the United States has been characterized by scientific talent training, rich and comprehensive content, a wide range of services, various implementation approaches, unique and effective methods, rapid research progress, standardized development of qualification certification, and a complete theoretical and practical system. According to the retrieval and analysis of relevant literature, in the early stages, the United States was mainly permeated by the curriculum of physical education and moral education, and there was no special mental health education curriculum [13, 14]. However, some schools will offer psychology courses such as introduction to psychology and social psychology in social subjects, mainly for students to better adapt to society and learn to use psychological theories to adjust to emotions and pressure. Among Asian countries, Japan is the first country to carry out school mental health education research. At present, Japan has formed a primary and secondary school health education network of one school, one community, and one family by the government, with a sound school psychological counseling mechanism and relevant laws and policies. Similar to the United States, the mental health education courses in Japanese schools are scattered and infiltrated with moral education, health care, sports, and other in-class activities, and there are no separate mental health education courses. The main occupation of students is learning. Because of the existence of competitive pressure, their psychological problems generally come from learning, so it is necessary to infiltrate the discipline of mental health education. There are many documents and papers in detail to discuss this point of view and put forward the significance of infiltration ways.

It is not difficult to see from the above content that there is some theoretical support for the penetration of psychological health education in discipline teaching. In recent years, some practical studies have shown that the penetration of mental health education into college courses can provide learners with opportunities to express their emotions and interact with each other, so as to improve the motivation level of the students and improve their individual autonomy. Take the United States as an example. We now gradually try to adopt the whole grade multidisciplinary curriculum infiltration mode and emphasize the common participation of teachers and students to achieve the purpose of mental health education [15, 16]. Compared with western countries, mental health education in China started late. School mental health education, as the most important, basic, and effective way to carry out mental health education in China, is the focus and starting point of Chinese scholars' research. The research on mental health education in foreign countries started earlier with rich theoretical achievements and practical experience. The research on the problems existing in the integration of mental health education into ideological and political education in colleges and universities has always been the focus of academic attention. Only by identifying the existing problems can we lay the foundation for putting forward targeted countermeasures. The academic circle is mainly summarized from three perspectives: educator, educated, and educational environment. To sum up, although the academic circle of mental health education in college teaching research results are quite abundant, the research quality is not high, and there are some deficiencies. The specific performance is as follows: first, the research on the relationship between the two is not in-depth enough, and some views remain superficial and persuasive. Second, there is a lack of systematic investigation and the process cannot be thoroughly grasped. Thirdly, many of them are discussed from a macro perspective, and the requirements proposed are not strong in implementation and lack innovation.

It is clearly pointed out in the teaching syllabus of the basic stage of French majors in colleges and universities that the teaching aim of the basic stage of French learning [17, 18] is to have the basic skills of listening, speaking, reading, and writing as well as certain communication skills, and have the preliminary self-learning ability, which will lay a good foundation for the improvement of French learning or other professional courses with French as a tool. The general idea of the syllabus for senior French majors in colleges and universities is consistent with the syllabus for the basic stage of French majors in colleges and universities, which places more emphasis on the cultivation of students' social and cultural knowledge and independent working ability. In terms of teaching principles, apart from strengthening the training of basic language skills, it is also required to expand the scope of students' knowledge, and it is pointed out that the imparting of language skills complements each other. To know the Francophone countries' social and cultural background, master the language and acquire knowledge related to professional orientation [19, 20]. Attention should be paid to the cultivation of students' ideological quality, the use of heuristics and discussion methods, and fully mobilize the initiative and enthusiasm of students to learn. To sum up, it can be seen that the overall requirements of the teaching syllabus for French majors in China are based on teaching students French language knowledge and training French language skills. The ultimate goal is to cultivate students' French communicative ability and organize and arrange teaching content according to social demand, students' employment tendencies, and the school's own characteristics. In the teaching process with students as the center, the use of heuristics and discussion teaching methods are adopted.

In terms of teaching methods, French teaching researchers have explored the perspectives of teaching AIDS, teaching models and methods, and the application of linguistics in teaching [21, 22]. The research covers a wide range of areas, and the content of the discussion is also more in-depth, which provides some specific ideas and references for the model, method, and means of French teaching in China. Since our country's French professional teaching content mainly focusses on imparting French language knowledge while ignoring the oral and listening training, especially the cultivation of student's French communicative competence, the consequences are many. The students scored better marks in grammar knowledge, but the poor performance problem in speaking and listening needs to solved. Some students have mastered the French language and have a certain listening and speaking ability, but they know little about French history and culture, local customs, social etiquette, oral habits, and so on. Their intercultural communication ability is relatively poor. Therefore, many French teaching researchers have made great efforts to change this situation and have conducted in-depth research and discussion on the contents of French teaching, including oral French teaching, French listening teaching, French culture teaching, and other aspects. At present, there are few studies on French learners in China, which mainly focus on learners' needs analysis, learners' psychological analysis, and learning effects evaluation [23, 24].

At present, most research on students' mental health problems uses questionnaires. With the rise of educational data mining, a few researchers use students' online behavior to identify students with mental health problems. In this paper, we will take a look at the current state of research on educational data mining [25, 26]. In the 20^th^ century, many colleges and universities at home and abroad began to use data mining technology to analyze educational data and introduced the concept of education data mining (EDM) [27, 28]. Their research aims to extract valuable information from educational data so that students can better complete their studies. The above studies illustrate the application of EDM in five aspects: grant issuance, career choice, changing trend and the gender difference in students' campus behavior, students' school performance, and students dropping out. In recent years, EDM has also been studied in the field of mental health issues, which will be described in detail in the next section. EDM is a direction worth exploring. Although there is still little research on EDM at present, with the explosive growth of network data and the increasingly sound construction of digital campuses, more valuable information will be mined from EDM, and the quality of education will be better in the future at this pace. At the same time, students' physical and mental health will be further improved. Therefore, this paper proposes a method of integrating mental health education and French teaching based on artificial intelligence technology [29, 30]. The main contributions of this paper are given as follows:

1. This paper is the first to integrate mental health education into French teaching in universities.
2. The research in this paper not only has good theoretical results but also has great potential application value.

## 3. The Proposed Integrating Mental Health Education into French Teaching Method

### 3.1. Machine Learning Method in EDM

Machine learning is a process in which computers are used. With computers learning patterns and patterns from massive amounts of data, machine learning can infiltrate useful information to solve some problems in life. Machine learning generally includes supervised learning, semisupervised learning, and unsupervised learning according to the type of task [31, 32]. When solving a problem, the target of the problem needs to be analyzed to select the appropriate type of machine learning. The goal of supervised learning is to learn the laws and patterns of a known dataset and build a model. The characteristics of the training set can be input into the model to obtain the corresponding output. When some new samples are input, the model can be used to obtain the corresponding output results. Depending on the different output results, supervised learning can be divided into regression (continuous value) and classification (discrete value). In unsupervised learning, all samples in a dataset are unlabeled. Its goal is to observe the interrelationship between data samples by analyzing hidden patterns in the data and dividing the dataset samples into different groups or clusters. In semisupervised learning, some samples in the dataset are labeled and some samples are unlabeled. The process is to train the model with a small amount of labeled data and a large number of unlabeled datasets and find out the rules.

The process of EDM is basically the same as that of data mining, mainly including the following steps [33, 34]: (1). Data collection: Due to different educational environments and systems, the data collected for solving different problems are also different. There are many sources of educational data, including management system data, psychological counseling data, and questionnaire data. It is very necessary to collect and sort out these multisource data. (2). Preprocessing: Educational data is complex and diverse. On the one hand, to solve the same problem, different education systems generally have different storage formats, so relevant data need to be extracted according to the actual problem. On the other hand, it is critical to extract the best data structure based on the type of problem being solved. So, converting the raw data into a suitable data structure can help solve the problem. (3). Data mining: Data mining technology is used to analyze educational data. In the field of education, data mining technologies such as classification, clustering, and association analysis are usually used. Finally, the educational environment or system can be improved according to the results of the experiment. For decision-making, we can interpret models derived from data mining algorithms and then design systems that provide decisions, opinions, or recommendations to relevant educators. This automated system saves educators both time and manpower.

### 3.2. BP (Back Propagation) Neural Network

The diagram of the BP neural network is given in Figure 1. The network training process is given as follows:

(1) $$\begin{array}{c} E=\sum_{i=1}^{m}{\left(x_{i}-c_{i}\right)}^{2}, \end{array}$$

where *x*_*i*_ is the input of the model, *c*_*i*_ is the bias of the model. And *m* is the number of the nodes, thus, the *E* is the training error of the model. Therefore, the training model can be iterated through cross-entropy loss. Model errors can be reduced through training and iteration to achieve the best model performance. Then, the hidden layer can be expressed:

(2) $$\begin{array}{c} E=\frac{1}{2}\sum_{\kappa =1}^{\ell }{\left[d_{\kappa }-f\left({\text{net}}_{\kappa }\right)\right]}^{2}=\frac{1}{2}\sum_{\kappa =1}^{\ell }{\left[d_{\kappa }-f\left(\sum_{j=0}^{m}\omega_{j\kappa }y_{j}\right)\right]}^{2}. \end{array}$$

When expanded further to the input layer, there is,

(3) $$\begin{array}{c} E=\frac{1}{2}\sum_{\kappa =1}^{\ell }d_{\kappa }-f\left[\sum_{j=0}^{m}\omega_{j\kappa }f\left({\text{net}}_{\text{j}}\right)\right]\\ =\frac{1}{2}\sum_{\kappa =1}^{\ell }d_{\kappa }-f{\left[\sum_{j=0}^{m}\omega_{j\kappa }f\left(\sum_{j=0}^{n}v_{ij}\chi_{i}\right)\right]}^{2}. \end{array}$$

It can be seen from the above formula that the network input error is a function of the weights of each layer, so the error can be changed by adjusting the weights. Obviously, the principle of adjusting weights is to reduce errors continuously, so the weights should be proportional to the gradient descent of errors.

(4) $$\begin{array}{c} \Delta \omega_{j\kappa }=-\eta \frac{\partial E}{\partial \omega_{j\kappa }}\\ j=0,1,2,\ldots ,m;\\ \kappa =1,2,\ldots ,\ell ,\\ \Delta v_{ij}=-\eta \frac{\partial E\partial }{v_{ij}}\\ i=0,1,2,\ldots ,n;\\ j=1,2,\ldots ,m. \end{array}$$

And weight adjustment process is,

(5) $$\begin{array}{c} \Delta \omega_{j\kappa }^{h+1}=\eta \delta_{h+1}^{\kappa }y_{j}^{h}=\eta \left(d_{\kappa }-o_{\kappa }\right)o_{\kappa },\\ \Delta \omega_{pq}^{1}=\eta \delta_{q}^{1}\chi_{p}=\eta \left(\sum_{r=1}^{m_{2}}\delta_{r}^{2}\omega_{qr}^{2}\right)y_{q}^{1}. \end{array}$$

The optimization algorithm proposed in this paper is used to optimize the parameters of BP neural networks so as to achieve the best model performance. The differential evolution algorithm (DE) is used to optimize the initial weights and thresholds of the network.

(6) $$\begin{array}{c} x_{i,1}=x_{i}^{L}+\mathrm{rand}\left(x_{i}^{U}-x_{i}^{L}\right),i=1,2,\cdots ,NP. \end{array}$$

The mutation operation can be expressed as follows:

(7) $$\begin{array}{c} v_{i,G+1}=x_{r1,G}+F\left(x_{r2,G}-x_{r3,G}\right),\\ u_{ji,G+1}=\left\{\begin{array}{cc} v_{ji,G+1} & r_{j}\leq CR\text{or}j=\mathrm{rand}\left(i\right),\\ x_{ji,G} & r_{j}\geq CR\text{or}j\neq \mathrm{rand}\left(i\right). \end{array}\right. \end{array}$$

Similar, the selection operations are denoted as follows:

(8) $$\begin{array}{c} x_{i,G+1}=\left\{\begin{array}{cc} u_{i,G+1} & f\left(u_{i,G+1}\right)\leq f\left(x_{i,G}\right),\\ x_{i,G} & f\left(u_{i,G+1}\right)>f\left(x_{i,G}\right). \end{array}\right. \end{array}$$

Following formula is a fitness function, the range is the entire set of real numbers.

(9) $$\begin{array}{c} f\left(X\right)=\sqrt{\frac{1}{N}\sum_{i=1}^{N}{\left(Y_{i}^{0}-Y_{i}\right)}^{2}}. \end{array}$$

Conventional BP neural networks cannot process complex psychological data online, especially when psychological education is integrated into French teaching in universities. Therefore, it is urgent to put forward an improved BP model to be suitable for the problem scenario in this paper.

### 3.3. The Framework of the Proposed Method

Based on the above discussions, the optimized BP neural network and its application in the analysis of the integration of mental health education into French teaching in universities are shown in Figure 2.

## 4. Experimental Results and Analysis

### 4.1. Data Collection and Experimental Environment

We surveyed 300 undergraduate students at a certain university, 250 of whom were assessed as having mental health problems by experts at the school's psychological center. In our experiment, students were divided into two categories: mild, moderate and severe. Students with mental health problems reflect positive samples, and students without mental health problems reflect negative samples.

The model needs real datasets in the process of training and testing, and datasets are generally divided into training sets and test sets. The training set is used in the training process of the model, and the parameters of the model can be adjusted through labels in the training sample. During the training process, the model will adjust parameters once for every training sample. The test set is used in the testing process of the model. The model can be evaluated by comparing the labels of the test samples with the predicted values. The whole process does not change any parameters. The details of the network model designed in this paper are shown in Figure 3. Although the structure of the BP model can be designed in many ways, the model design chosen for this article is shown in Figure 3, mainly because it can achieve the best results under these settings.

### 4.2. Experimental Results Analysis

During model training, the model accuracy and loss change increase as the number of iterations increases, as shown in Figure 4, where the horizontal coordinate is the number of iterations, the vertical coordinate is the loss value, and the horizontal and vertical coordinates are dimensionless values, so they have no units. With the increase in iteration times, the model loss becomes smaller and tends to be stable. When the number of iterations is 40, the loss of the model tends to be stable. Therefore, we set the number of iterations to 40. From the results of the visualization model, the whole training process is relatively stable, which shows the stability and practicability of the method presented in this paper.

Because the performance of a model can be characterized by many indicators, it is difficult to apply all indicators in one article. Therefore, only RMSE, precision, and recall are used in this paper to describe the performance of the proposed method because these three indicators can comprehensively describe the performance of the model from multiple angles. In order to further verify the effectiveness of the method, the performance comparison of different methods is presented in Figure 5, in which convolutional neural networks and conventional BP neural networks are selected as the comparison algorithms. Precision is the predicted results against us. It represents the prediction of samples as to how many samples are true. The recall rate is according to our original sample. The samples predicted correctly is the denominator. The denominator is right in the prediction of the number of samples. The other one is the original sample of all of the samples. From the figure we know, the DE-BP obtained the highest recall and precision result. Though the RMSE (Root Mean Square Error) is a little higher than the contrast method, it is well within the acceptable range, at about 1.7. It is worth noting that although the CNN model is a deep learning method, its model performance is still worse than DE-BP, mainly because the DE-BP model obtains the best model parameters through an optimization algorithm, so as to achieve the best model effect. This means achieving the highest recall and precision values.

In order to show the influence of the proposed mental health education method on the mental health levels of male and female students, Figure 6 shows the changes in mental health over time. As can be seen from the figure, with the passage of time, the mental health level of all students presents the above trend, indicating that the proposed DE-BP-based mental health feature extraction method is effective. However, the rising level of boys is significantly higher than that of girls, mainly because boys may have a stronger acceptance ability or psychological ability to resist pressure. It is worth noting that Figure 6 shows the development and change of male and female mental health levels during college years. Hence, the horizontal and vertical coordinates of Figure 6 are dimensionless values; that is, they have no units.

Furthermore, Figure 7 shows the test results of abnormal mental health conditions of students in different grades. Blue, purple, green, and black represent freshmen, sophomores, juniors, and seniors. As can be seen from the graph, the frequency of psychological abnormalities is increasing with the increase in students' grades. It is worth noting that the curves in different colors in Figure 7 represent different grades. Since there are only four grades in the college, there are only four color curves in this figure.

Finally, Figure 8 shows the change in French teaching effects before and after the integration of mental health education. Different colors in the figure represent different French abilities. It can be seen from the figure that different French learning abilities have been improved to different degrees after the integration of mental health education, thus demonstrating the promotion effect of integration of mental health education on French teaching in universities. Therefore, the reliability and practicability of the proposed method are further illustrated. It is worth noting that k on the ordinate in Figure 8 represents units of people, i.e., thousands. Therefore, the larger the ordinate is, the more people are involved in the improvement of the French teaching effect, which indicates that the method in this paper is more effective. Thus, the right side of Figure 8 demonstrates the validity of the proposed method.

## 5. Conclusion

This study clarified the present research status of the infiltration of French teaching by sorting out and analyzing literature and materials and it believed that it was very important to conduct further research on the infiltration of French teaching into mental health education after the core quality of French discipline was proposed. This study investigated the present situation of the integration of French teaching and mental health education in front-line universities and used the improved BP neural network to analyze and evaluate the psychological data and apply it to teaching practice to test the effectiveness of the strategy. Although the method in this paper has achieved good performance, it is still a lightweight deep model. Thus, in the face of big data scenarios, the proposed method is not enough, and a depth-based method to integrate mental health education into French teaching will be the focus of future research.

## Figures and Tables

**Figure 1:** The diagram of the BP neural network.

**Figure 2:** The model structure diagram of the proposed method.

**Figure 3:** The BP neural network structure designed in this paper.

**Figure 4:** The relationship between epoch and loss during training.

**Figure 5:** Comparison of model performance between different methods.

**Figure 6:** The development and change of male and female mental health levels during college years.

**Figure 7:** The psychological abnormalities of different grades in the college.

**Figure 8:** Comparison of French teaching effects.

## Data Availability

The datasets used during the current study are available from the corresponding author on reasonable request.
